# Dual-Path Attention Compensation U-Net for Stroke Lesion Segmentation

**DOI:** 10.1155/2021/7552185

**Published:** 2021-08-31

**Authors:** Haisheng Hui, Xueying Zhang, Zelin Wu, Fenlian Li

**Affiliations:** College of Information and Computer, Taiyuan University of Technology, Taiyuan 030024, China

## Abstract

For the segmentation task of stroke lesions, using the attention U-Net model based on the self-attention mechanism can suppress irrelevant regions in an input image while highlighting salient features useful for specific tasks. However, when the lesion is small and the lesion contour is blurred, attention U-Net may generate wrong attention coefficient maps, leading to incorrect segmentation results. To cope with this issue, we propose a dual-path attention compensation U-Net (DPAC-UNet) network, which consists of a primary network and auxiliary path network. Both networks are attention U-Net models and identical in structure. The primary path network is the core network that performs accurate lesion segmentation and outputting of the final segmentation result. The auxiliary path network generates auxiliary attention compensation coefficients and sends them to the primary path network to compensate for and correct possible attention coefficient errors. To realize the compensation mechanism of DPAC-UNet, we propose a weighted binary cross-entropy Tversky (WBCE-Tversky) loss to train the primary path network to achieve accurate segmentation and propose another compound loss function called tolerance loss to train the auxiliary path network to generate auxiliary compensation attention coefficient maps with expanded coverage area to perform compensate operations. We conducted segmentation experiments using the 239 MRI scans of the anatomical tracings of lesions after stroke (ATLAS) dataset to evaluate the performance and effectiveness of our method. The experimental results show that the DSC score of the proposed DPAC-UNet network is 6% higher than the single-path attention U-Net. It is also higher than the existing segmentation methods of the related literature. Therefore, our method demonstrates powerful abilities in the application of stroke lesion segmentation.

## 1. Introduction

Recent global statistics on the incidence of stroke cases demonstrate that there are up to 10.3 million new cases annually [1]. Stroke has become one of the top three lethal diseases, besides chronic diseases. When a stroke occurs, accurate diagnosis of the severity of the stroke and timely thrombolytic therapy can effectively improve blood supply in the ischemic area and significantly reduce the risk of disability or even death. Therefore, it is clinically significant to quickly and accurately locate and segment the stroke lesions [2]. Since manual segmentation relies on the doctor's professional experience and medical skills, individual subjectivity can reduce segmentation accuracy. Furthermore, manual segmentation of the stroke lesion is time-consuming. It may take a skilled tracer several hours to complete accurate labeling and rechecking of a single large complex lesion on magnetic resonance imaging (MRI) [3].

This situation has changed after the advent of convolutional neural network (CNN) [4] and its continuously evolving network structures, such as fully convolutional network (FCN) [5] and SegNet [6], which have achieved success in the field of image segmentation, especially medical image segmentation [7]. However, CNN-based segmentation networks require a large amount of labeled medical data for training, which is limited by the high cost of acquiring and accurate labeling [8]. The multilevel U-shaped network (U-Net) [9] based on CNN, consisting of the contraction and expansion paths, mitigates the problem of requiring huge amounts of labeled data. The U-Net network structure and its improved network structure, such as the attention U-Net [10], U-Net++ [11], and R2U-Net [12], have been applied successfully in medical segmentation tasks, such as skin cancer [13], brain tumor [14], colorectal tumor [15], liver [16], colon histology [17], kidney [18], and vascular borders [19]. The U-Net network has thousands of feature channels, especially the standard U-Net model with a five-level structure with enormous parameters to be trained. During the training process, the contraction path (encoder) and expansion path (decoder) need to repeatedly extract deep-scale features. The deep-scale features of standard U-Net are considered abstract and low-resolution features, which increase the training difficulty and make the training unstable and inadequate.

To reduce the training difficulty caused by repeated extraction of deep-scale features and improve segmentation accuracy, many researchers employed a two-step method to locate the lesion and segment the target area [20, 21]. However, these methods introduce additional positioning operations and cannot achieve end-to-end training. Schlemper et al. introduced a self-attention mechanism and proposed an attention U-Net with an attention gate (AG) [10] to avoid additional operations. The self-attention mechanism reduces the dependence on external information obtained from additional steps by utilizing the correlation coefficient of feature signals from different scales. This mechanism captures the internal correlation of features and focuses attention on the target area. The attention U-Net uses AG to generate a 2D attention coefficient map to suppress irrelevant regions in an input image while highlighting salient features useful for specific tasks. The AG module can be integrated into the standard U-Net model for end-to-end learning without additional pretraining steps. Compared with the standard U-Net training parameters, the number of training parameters slightly increased with additional computation of AG operations. The use of the built-in self-attention module eliminates the use of additional target location operations. It achieves the goal of reducing training difficulty, improving training efficiency, and improving model segmentation performance.

However, the self-attention mechanism based on correlation operation has some deficiencies. The attention coefficient *α* for constraining the area of interest is generated by the current-scale feature signal *x* and the rougher-scale feature signal *g* derived from *x*, leading to a potential risk of the segmentation network using the self-attention mechanism. It implies that a small lesion with a nondistinct lesion feature may cause the current level feature signal *x* to learn the lesion feature inadequately. Consequently, the deviation of the attention area from the lesion area due to the wrong or insufficient attention coefficient learning leads to incorrect segmentation results.

To solve the problem of the attention area deviating from the lesion area, we proposed a dual-path attention compensation U-Net (DPAC-UNet) network, which is composed of the primary path network (primary network) and auxiliary path network (auxiliary network). Both networks are all attention U-Net segmentation models based on the self-attention mechanism with an identical structure. The primary network is the core part of DPAC-UNet, which performs lesion segmentation and outputs the final segmentation result. The auxiliary network is used to generate an auxiliary attention compensation coefficient map sent to the primary network to compensate for possible attention coefficient learning errors. The auxiliary network realizes its compensation ability by focusing on a larger area than the actual lesion area, which increases the coverage of the attention coefficient map generated by the auxiliary network. The attention coefficient map with a larger attention area is defined as a tolerant attention coefficient map, which is used as an auxiliary compensation attention coefficient to compensate for possible errors in the primary network attention coefficient map. To study our lesion segmentation network, we use the ATLAS dataset [3], consisting of 239 T1-weighted subacute and chromic stroke MRI scans released in 2018.

The main contributions of this article are summarized as follows:

1. We proposed a DPAC-UNet that uses the auxiliary network to generate an attention coefficient map with a larger area to compensate for the possible defect of the primary network's attention coefficient map.
2. We proposed the WBCE-Tversky loss and tolerance loss to train the primary and auxiliary networks of the DPAC-UNet to realize their effects on the entire network, respectively, and explore the optimal hyperparameter configurations of the two proposed loss functions.

The remainder of this work is organized as follows: In Section 2.1, we describe the network structure of the DPAC-UNet and how to use the auxiliary network to compensate for attention in the primary network.  Section 2.2 proposes two compound loss functions, the WBCE-Tversky loss and the tolerance loss. In this section, we also conducted experiments to discuss the effect of different hyperparameter values of the loss functions on the performance of the segmentation task. Finally, the steps to select the optimal hyperparameter configuration of the two proposed loss functions are listed. In Section 3, we train the DPAC-UNet by the WBCE-Tversky and the tolerance loss functions with the optimal hyperparameter configurations. In this section, a visualization example is also presented to demonstrate the effectiveness of the DPAC-UNet network further. We also discussed the time consumption of the primary and auxiliary networks of the DPAC-UNet, and we also tried to execute the auxiliary network's compensation mechanism for other segmentation models with self-attention mechanisms.

## 2. Materials and Methods

### 2.1. DPAC-UNet

The attention U-Net introduces several attention gates (AG) to generate attention coefficient maps that suppress irrelevant regions in an input image while highlighting salient features useful to improve segmentation performance without introducing additional positioning operations. However, it sometimes makes mistakes. A small lesion with indistinct lesion features is difficult to distinguish from the surrounding healthy tissues, leading to the current scale feature signal *x* of a certain layer not learning the lesion feature well. As a result, the attention coefficient generated using *x* and its derived rougher feature *g* will deviate from the lesion area. Therefore, the wrong attention coefficient results in the AG outputting the wrong feature signal, which affects the segmentation results. Thus, if the attention U-Net finds the correct lesion in the AG module, it will emphasize the relevant area and suppress the unrelated area to improve the segmentation performance. Conversely, if the lesion location is not found in the AG or is wrong, it will result in diametrically opposite effects and degrade the segmentation performance. To cope with the previously mentioned issues, using the attention U-Net as the basic segmentation model, we propose the DPAC-UNet network.

#### 2.1.1. Overview of the Structure

The schematic of DPAC-UNet is presented in Figure 1. We used two identical attention U-Net models as the primary and auxiliary network segmentation models, which correspond to the upper and lower half of Figure 1, respectively. The WBCE-Tversky loss function trains the primary network for accurate segmentation. The auxiliary network is trained by the tolerance loss to generate a tolerant auxiliary compensation attention coefficient that compensates for the defect of the attention coefficient map of the primary network. The details of the two loss functions are described in Section 2.2. As presented in Figure 1, the auxiliary network compensates for the auxiliary compensation attention coefficient to the primary network through the vertical dark red arrow line from the AG marked (II) to the AG marked (I), in order to perform the compensation operation. We just selected the second-level AG of the primary and auxiliary networks for additive compensation operation. This is because the resolution of the attention coefficient maps generated by the two bottom AGs (13 × 11 and 26 × 22) is too low. The difference between the attention maps of the two networks on this resolution scale is larger due to the difference of one pixel. When the level is deeper, the receptive field affected by a single pixel is very large. Consequently, the compensation operation at this scale by the auxiliary network has a significant impact on the primary network, and the compensating operation generates a significant attention fluctuation. Furthermore, the first-level AG, which is close to the uppermost layer's output, does not perform auxiliary attention compensation operation because the feature map here is too close to the output and affects the segmentation result. In summary, we only selected the second-level AG to implement the compensation operation in order to effectively compensate for the defective attention coefficient map of the primary network and ensure that it does not directly affect the accuracy of lesion segmentation of the primary network.

Figure 2 presents the AG schematic of the primary and auxiliary networks at the second level. The AG of the first, third, and fourth levels are shown in Figure 1, which are not involved in auxiliary attention coefficient compensation operation and are identical in structure to the AG in the literature [10]. The AG marked as (II) in the lower half of Figure 1 is the second-level AG in the auxiliary network's attention U-Net, and its detailed structure is shown in Figure 2(a). In Figure 2(a), ① and ② are the input of the auxiliary network AG, ④ is the output of the current level for skip connection (SC), where *l* is the level number of current AG (in this case *l*=2), and feature signals *x*_*i*_^*l*^ and *g*_*i*_^*l*^ correspond to the inputs labeled ① and ②. The feature signals *g*_*i*_^*l*^ ∈ *R*^*F*_*g*_^ and *x*_*i*_^*l*^ ∈ *R*^*F*_*x*_^ are sent to the AG block to generate the attention coefficient *α*^*l*^ using the additive attention generation operation in order to determine the area to focus, where *i* is the pixel number,*F*^*x*^ is the number of feature channels of input feature signal *x*^*l*^ at the current level, and*F*^*g*^ is the number of feature channels of input feature signal *g*^*l*^ at the rougher level. When the additive attention coefficient map *α*^*l*^ is generated using *x*_*i*_^*l*^ and *g*_*i*_^*l*^, the feature signal *x*_*i*_^*l*^ is multiplied by *α*^*l*^ and used as the output of the AG gate and sent to the decoding path through the SC at the current level. The additive attention coefficient *α*^*l*^ marked as ③ is the auxiliary compensation attention coefficient map and sent to the AG marked as (I) at the same level and in the same position of the primary network in the upper half of Figure 1. The equations for generating the attention coefficient of the auxiliary network are as follows:

(1) $$\begin{array}{c} q_{att}^{l}=W_{\psi }^{T}\left(\sigma_{1}\left(W_{x}^{T}x_{i}^{l}+W_{g}^{T}g_{i}^{l}+b_{g}\right)\right)+b_{\psi }, \end{array}$$

(2) $$\begin{array}{c} \alpha_{i}^{l}=\sigma_{2}\left(q_{\text{att}}^{l}\left(x_{i}^{l},g_{i}^{l};\Theta_{\text{att}}\right)\right), \end{array}$$

(3) $$\begin{array}{c} {\left(\alpha_{i}^{l}\right)}_{rs}=\text{resample}\left(\alpha_{i}^{l}\right), \end{array}$$

(4) $$\begin{array}{c} \hat{x_{i}^{l}}=x_{i}^{l}\cdot {\left(\alpha_{i}^{l}\right)}_{rs}. \end{array}$$

As presented in Figure 2(a), considering the inconsistent spatial resolution and feature channel dimensions of feature *g*_*i*_^*l*^ and *x*_*i*_^*l*^, we also need to use the upsampling operation to change the spatial resolution of the signal *g*_*i*_^*l*^ to make it consistent with *x*_*i*_^*l*^. Moreover, we need to use the linear transformation *W*_*g*_ ∈ *R*^*F*_*g*_×*F*_int_^ and *W*_*x*_ ∈ *R*^*F*_*x*_×*F*_int_^ to make the number of feature channels of these two signals the same, where *b*_*g*_ ∈ *R*^*F*_int_^ and *b*_*ψ*_ ∈ *R* denote the biases of the two linear transformations. In (1), *σ*_1_ is the ReLU activation function, and the output of this activation function is linearly transformed by *W*_*ψ*_^*T*^ ∈ *R*^1×*F*_int_^ that forms an attention coefficient matrix with only one feature channel. In (2), the sigmoid activation function *σ*_2_ converts the attention coefficient matrix into a gridded attention coefficient map *α*_*i*_^*l*^ to act on *x*_*i*_^*l*^. Resample *α*_*i*_^*l*^, and then, multiply the resampled result by *x*_*i*_^*l*^ to generate the AG output feature signal ${\hat{x}}_{i}^{l}$.  Figure 2(b) presents the block diagram of the AG marked as (I) in the upper half of Figure 1, where the auxiliary compensation attention coefficient map compensates for the primary network. The structure and equations of the signal operation process are almost consistent with the auxiliary network, as presented in Figure 2(a). The difference is that when generating the final additive fused attention coefficient map, the auxiliary compensation attention coefficient map generated by the auxiliary network AG is marked as ③, and perform additive fusion together with the original attention coefficient map generated by the primary network AG generated by inputs ① and ②. According to (3) and (4), the output feature signal ④ of the primary network AG is generated.  Figure 2(c) presents the definition of various operation symbols and dimension changes of input and output feature signals in Figures 2(a) and 2(b).

#### 2.1.2. Compensation Mechanism of the Auxiliary Network

The traditional single-path self-attention model generates a spatial attention coefficient map by the AG to cover the lesion area of features to pay more attention to the lesion area to improve the segmentation performance. Our proposed method builds an auxiliary network to generate an auxiliary attention coefficient map with a larger coverage area to compensate the segmentation network (primary network) to improve its hit rate of complete coverage of the lesion by spatial attention coefficient map. It should be noted that the attention compensation map will not deviate from the original attention area of the primary network but will be constrained to increase the attention area around it. This compensation mechanism is especially effective when the lesion feature is indistinct, the lesion's outline is unclear, or the segmentation model cannot generate the correct region of interest.

The qualitative analysis and comparison of using the primary network individually or combined with an auxiliary network are stated as follows. When DPAC-UNet uses the auxiliary network to compensate for the primary network, there are three situations:

 
*Situation 1.* (1) Use the primary network individually: when the focus area of the attention coefficient map of the single-path network is partially correct (Figure 3(a), ①), which will lead to reduced segmentation performance. (2) Combined with an auxiliary network: after the auxiliary network compensates the primary network's attention coefficient map with a larger focus area through additive compensation, the compensated attention coefficient map may be correct (Figure 3(a), ②) or remain unchanged (Figure 3(a), ③), which will eventually improve the segmentation performance or maintain the segmentation performance.
 
*Situation 2.* (1) Use the primary network individually: when the focus area of the attention coefficient of the primary network is completely correct, which will generate correct segmentation results (Figure 3(b), ①). (2) Combined with an auxiliary network: although the auxiliary network compensates it for a larger attention coefficient map, after the addition compensation operation, the value of the original correct focus area becomes larger, and the values of other areas are still smaller than the value of the correct area (Figure 3(b), ②). Therefore, the primary network of DPAC-UNet can still pay higher attention value in the correct area and keep the segmentation performance unchanged.
 
*Situation 3.* (1) Use the primary network individually: when the focus area of the primary network attention coefficient is completely wrong (Figure 3(c), ①), which will lead to reduced segmentation performance. (2) Combined with an auxiliary network: the larger auxiliary attention coefficient compensation map generated by the auxiliary network covers a larger area, and the compensated attention coefficient map may be still wrong (Figure 3(c), ②), or correct partially (Figure 3(c), ③), or correct completely (Figure 3(c), ④). At this time, correspondingly, the segmentation performance will remain unchanged, or improve to some extent, or improve significantly.

Therefore, by combining the previously mentioned three situations, the overall average segmentation performance of the whole dataset will be improved. It can also be seen from Figure 3 that the attention coefficient map generated by the auxiliary network does not deviate from the attention coefficient map area generated by the primary network.

### 2.2. Loss Functions of DPAC-UNet

We proposed two different compound loss functions to train the primary and auxiliary networks. First, we proposed the WBCE-Tversky loss for the primary network to generate an attention coefficient map focused on the target area and an accurate segmentation result. Second, we proposed the tolerance loss for the auxiliary network to generate an auxiliary compensation attention coefficient map with a larger coverage area to compensate for the primary network. It is called a tolerance loss because it can generate an attention coefficient map that covers a larger area and does not deviate from the lesion area, which means a higher fault tolerance for attention errors.

#### 2.2.1. WBCE-Tversky Loss

The Tversky loss [22], which was proposed to address data imbalance in medical image segmentation, is introduced as a component of our WBCE-Tversky. The Tversky loss is as follows:

(5) $$\begin{array}{c} T_{\text{loss}}\left(\alpha ,\beta \right)=1-\frac{\sum_{i=1}^{N}p_{1}i\cdot g_{1}i}{\sum_{i=1}^{N}p_{1}i\cdot g_{1}i+\alpha \sum_{i=1}^{N}p_{1}i\cdot g_{0}i+\beta \sum_{i=1}^{N}p_{0}i\cdot g_{1}i}, \end{array}$$

where *p*_1,*i*_ denotes the probability that a voxel is a lesion and *p*_0,*i*_ denotes the opposite, and *g*_1,*i*_ denotes the probability of whether a voxel is a lesion and *g*_0,*i*_ denotes the opposite. The Tversky loss achieves a trade-off between false positives (FP) and false negatives (FN) by configuring the value of its hyperparameter *β* and *α*, where *α*+*β*=1. A higher *β* value implies that the trained model's *recall* is given greater weight than the precision, and the network pays more attention to FN. Often, the volume of the lesion is significantly smaller than that of healthy tissue. For example, in the 239 MRI scans of the ATLAS dataset, the voxel number ratio of the lesion to the background is about 3 : 1000. The high ratio of the nonlesion to lesion makes the segmentation network prone to focusing on the nonlesion area, therefore, predicting the lesions as nonlesions and increasing FN in the predicted results. To solve this problem, we increased the value of the hyperparameter *β* of Tversky loss. Larger *β* gives greater weight to *recall* than *precision* by placing more emphasis on FN. We assume that using higher *β* in our generalized loss function in training will lead to higher generalization and improved performance for the imbalanced dataset. So, we use the Tversky loss with higher *β* as a part of the WBCE-Tversky loss for training the primary network of DPAC-UNet. Meanwhile, in the tolerance loss, we also need to use a Tversky loss function to constrain the growth of the attention coefficient map to ensure that the larger and more tolerant focus area will not deviate from the lesion area. To compare the segmentation performance of the Tversky loss with the different hyperparameter values of *β* and select the appropriate hyperparameter *β* for the WBCE-Tversky loss and tolerance loss, we used the Tversky loss for the training the basic segmentation model, attention U-Net. The hyperparameter *β* of the Tversky loss ranges from 0.5 to 0.95, using 0.5 as the value interval. We conducted an experiment using the sixfold cross-validation, which is often used to train a model in which hyperparameters need to be optimized. We split the 239 stroke MRI scans into training, validation, and test sets by sixfold cross-validation according to Figure 4.

First, in each fold, we divided the data into training and test sets using a ratio of about 5 : 1 (199 : 40), and we ensured that all MRI scans of all test sets are not repeated. Second, we further split the training set in each fold into the inner training and validation sets using a ratio of about 4 : 1 (160 : 39). The validation set is used to select the best-performing model trained by the training set. Moreover, we also ensured that the training, validation, and test sets of each fold have the same lesion volume distribution for the accuracy of the experiment results. The lesion size distribution of fold 1 is presented in Figure 5.

The experimental configuration and results of training the attention U-Net using Tversky are presented in Table 1. We used 10 different *β* values to perform sixfold cross-validation and computed the average metric scores of all test sets' results. We used the dice similarity coefficient (DSC), F2 score (F2), precision (PRE), and recall (RE) as the metrics for the model evaluation. DSC is a widely used metric for evaluating the performance of the models; F2 score is often used to evaluate the performance of the models for imbalanced data; PRE quantifies the number of positive class predictions that belong to the positive class; RE quantifies the number of positive class predictions made out of all positive examples in the dataset. The experimental results of training the attention U-Net with different hyperparameter *β* values for the Tversky loss are presented in Table 1.

As presented in Table 1, the maximum RE value is obtained when *β* takes a large value of 0.95, and the maximum PRE value is obtained when the minimum value of 0.05 is taken. DSC and F2 scores reached the maximum when *β*=0.80. Simultaneously, a trade-off between PRE and RE has been made, indicating that, for the imbalanced ATLAS dataset, training a model using the Tversky loss with hyperparameter *β*=0.80 improves the segmentation accuracy. We need a loss function that can train the primary network of the DPAC-UNet to achieve an accurate segmentation. To improve the segmentation performance, we can handle the imbalanced dataset by selecting the hyperparameter *β* value of the Tversky loss to train the basic segmentation model in order to reduce the tendency of the lesion to be classified as nonlesion. As presented in Table 1, the use of the Tversky loss with hyperparameter *β*=0.80 to train the attention U-Net on the ATLAS dataset achieves the highest segmentation performance. However, as presented in (5), if the denominator of the Tversky loss is a small value, it causes instability in backpropagation and derivation. To solve this problem, we introduced the WBCE loss [23] as another part of the WBCE-Tversky loss. On the one hand, it avoids the problems of backpropagation and gradient calculation instability caused by the Tversky loss for small denominators. On the other hand, using the WBCE loss and giving greater weight to the minority class in the equation adapts to the imbalance of dataset and further improves the overall segmentation performance. The WBCE loss function has differentiable properties, which simplifies the optimization process. The equation of the proposed WBCE-Tversky loss is presented in (8). The compound loss function is composed of the Tversky loss (*β*=0.80) and WBCE loss, and their respective equations are presented as

(6) $$\begin{array}{c} {\text{WBCE}}_{\text{loss}}=-\frac{1}{N\sum_{i=1}^{N}wg_{n}}\log\left(p_{n}\right)+\left(1-g_{n}\right)\log\left(1-p_{n}\right), \end{array}$$

(7) $$\begin{array}{c} w=\frac{N}{\text{smooth}.+\sum_{n}g_{n}}, \end{array}$$

(8) $$\begin{array}{c} \text{WBCE}-\text{Tversky}={\text{WBCE}}_{\text{loss}}+T_{\text{loss}}\left(\beta =0.8\right). \end{array}$$

The WBCE loss adds weight *w* to the standard BCE loss to give the pixels more importance, and a higher training weight when the area of the lesion is small, thereby improving the segmentation performance for unbalanced datasets. As presented in (6), the main part of the WBCE loss is the same as the BCE loss [23]. The only difference is that we modified the calculation method of the weight *w* as presented in (7) and took the reciprocal of the proportion of lesion pixels to all pixels as the weight *w*, where *N* denotes the number of pixels in the entire image to be segmented and ∑_*n*_*g*_*n*_ is the number of lesion pixels to be segmented, andsmooth=1 is used to prevent division by zero error.

To test and verify the proposed WBCE-Tversky loss, we conducted a series of comparative experiments using the WBCE loss, Tversky loss with different hyperparameter *β*, and WBCE-Tversky loss with different *β*. The model used in the experiment, the experiment datasets, and the experiment conditions are the same as the experiments corresponding to Table 1. The experiment parameter configuration and results are presented in Table 2. As can be seen from Table 2, for the same hyperparameter *β*, the DSC and F2 scores of the WBCE-Tversky loss are better than that of the Tversky loss. The WBCE-Tversky loss also performs best at *β*=0.80. Compared with the WBCE loss, the segmentation accuracy improved significantly, the DSC score improved by 6.5%, and the F2 score increased by 12.5%. In summary, on the imbalanced ATLAS dataset, using the WBCE-Tversky loss with *β*=0.80 to train the attention U-Net model achieves the best segmentation performance. Therefore, we used WBCE-Tversky loss with *β*=0.80 as the loss function of the DPAC-UNet's primary network for accurate lesion segmentation.

#### 2.2.2. Tolerance Loss

When the focus area is larger than the actual lesion area, the FP of the model segmentation result increases. The FP and FPR are proportional, implying that we can indirectly measure the tolerant degree of the lesion area using FPR. To indirectly measure the tolerant degree of the auxiliary compensation attention coefficient map, we used the FPR value as an indicator to determine the tolerant degree of attention coefficient generated by the auxiliary network. To provide the primary network with a more tolerant auxiliary compensation attention coefficient map and a much larger coverage area, we proposed the tolerance loss by introducing a *specificity reducing item* combined with the Tversky loss. It is called tolerance loss because the compound loss function's training goal is to obtain an attention coefficient map with high tolerance. The proposed tolerance loss is presented in (11), where *S*_loss_(*λ*, *δ*) denotes the *specificity reducing item* presented in (10). The concept of *specificity reducing item* is based on the adjustment of *specificity*, which measures the proportion of negatives that are correctly identified, and *s* is presented in

(9) $$\begin{array}{c} \text{specificity}=\frac{\text{TN}}{\text{TN}+\text{FP}}, \end{array}$$

(10) $$\begin{array}{c} S_{\text{loss}}\left(\lambda ,\delta \right)=\lambda {\left(\frac{\sum_{i=1}^{N}p_{0}i\cdot g_{0}i}{\sum_{i=1}^{N}p_{0}i\cdot g_{0}i+\sum_{i=1}^{N}p_{1}i\cdot g_{0}i}-\delta \right)}^{2}, \end{array}$$

(11) $$\begin{array}{c} T_{\text{loss}}=S_{\text{loss}}\left(\lambda ,\delta \right)+T_{\text{loss}}^{2}\left(\beta =0.8\right). \end{array}$$

Generally, the nonlesions in the imbalanced dataset occupy a large part of the total area. Using the ATLAS dataset as an example, the *specificity* of the segmentation results is reached as high as 95%. Since FPR=1 − Specificity, it implies that the larger the proportion of nonlesions identified as nonlesions, the smaller the FPR, and the less tolerant the auxiliary compensation attention coefficient map. Therefore, we introduce a *specificity reducing item* to reduce the *specificity* of segmentation results, increase the FPR of the auxiliary network's training results, and increase the size of the coverage area of the attention coefficient map. As presented in (10) and (11), we used the hyperparameters *λ* and *δ* to control the weight of the *specificity reducing item* in the tolerance loss. We squared the *specificity reducing item* and the Tversky loss to balance the equation to make the backward derivation and backpropagation easier.

In (10), the *specificity reducing item* is the square of the difference between the *specificity* equation and *δ*. Since the training goal of any loss function is to make the value as small as possible, the training goal of (10) is to make value 0, which means that the value of *specificity* is close to the value of hyperparameter *δ*. Therefore, setting a reasonable *δ* can control the specificity value to the desired degree. The smaller the *δ*, the smaller the *specificity* obtained by the network training. As mentioned earlier, since FPR=1 − Specificity, the smaller the *specificity*, the larger the obtained FPR value, and the resulting attention coefficient map is more tolerant with a larger coverage area. We set the hyperparameter *δ* value of our tolerance loss to 0.6, 0.7, 0.8, or 0.9. The other hyperparameter *λ* is set to 1, 2, 3, 4, or 5 to adjust the contribution of the *specificity reducing item* of the tolerance loss. The value of the hyperparameter *β* is set to 0.8 according to the conclusion discussed in Section 2.2.1. The experiment results are presented in Table 3.

As presented in Table 3, the different FPR values generated by the tolerance loss with different hyperparameters *λ* and *δ*are compared. Based on (10), when *λ*=5, the tolerance loss gives the most significant weight to the *specificity reducing item*. Increasing *λ* and keeping *δ* constant produce higher FPR. Furthermore, the smaller the value of *δ*, the smaller the value of *specificity*, and the higher the FPR. In Table 3, the largest FPR value was obtained when *λ*=5, *δ*=0.6, and the FPR reaches as high as 18.97%. We also introduce a Tversky loss part to constrain the spatial position and contour shape of the lesion and restrict the growth of the attention coverage area with a high FPR value, rather than randomly increasing the FPR of the results.

As visual examples, we export the attention coefficient heatmaps of four MRI slices of different lesion sizes, which were segmented by the attention U-Net trained by tolerance loss with 10 varying configurations of hyperparameter. The attention coefficient heatmaps are generated by the AG (marked as II) in the auxiliary network in Figure 1. Note that, in the tolerance loss, the hyperparameter *β*=0.8 is fixed, because we used the other two parameters to adjust the FPR value. Considering the FPR of some values may be caused by a smaller *λ* and a larger *δ* or by a larger *λ* and a smaller *δ*, to draw the heatmaps, we sorted the FPR values in Table 3 and evenly selected 10 hyperparameter configurations of the tolerance loss according to the different FPR values. The attention coefficient heatmaps from the selected 10 hyperparameter configurations from Table 3 are also presented in Figure 6. It can be seen that as the FPR value increases, the coverage area of the attention coefficient map gradually increases. Due to the restriction of the Tversky loss part in the tolerance loss, although the focus area increased gradually, it did not deviate from the lesion area. Therefore, when tolerance loss is used in the auxiliary network of the DPAC-UNet, the primary network gets a compensation attention coefficient with the correct region irrespective of the increase of the FPR value and the coverage area. However, for the coverage area of the auxiliary compensation attention coefficient map, the case is not the larger the better, indicating that FPR is not as high as possible. We need to set a moderate value of hyperparameters *λ* and *δ* to provide the best segmentation performance for DPAC-UNet. Therefore, in Session 3, the optimal *λ* and *δ* hyperparameters will be selected based on the DPAC-UNet model depending on the experiment performance.

#### 2.2.3. Hyperparameter Selection

In order for the auxiliary network to generate a larger proper attention coefficient map, it needs to be trained by the tolerance loss proposed. Only when the hyperparameter configuration of the tolerance loss function is selected appropriately, the auxiliary network can provide moderate compensation to the attention module of the primary network to improve the segmentation performance. The selection process of loss function hyperparameter configuration of the primary and auxiliary network follows the following two steps:

 
*Step 1.* With 0.05 as the interval, from 0.5 to 0.95, using 10 different *β* values of Tversky loss to train the single-path Attention U-Net model, take the *β* value with the best segmentation performance as the selected *β* value of the proposed WBCE-Tversky loss and Tolerance loss.
 
*Step 2.* To select appropriate *δ* and *λ* values for the tolerance loss, so that the auxiliary network can provide appropriate attention coefficient map compensation and achieve the best segmentation performance of the entire DPAC-UNet, we use the WBCE-Tversky loss function (fix the *β* value that has been selected in the first step) to train the primary network. We set the tolerance loss *δ* value to 0.6, 0.7, 0.8, or 0.9, and set *λ* value to 1, 2, 3, 4, or 5; that is, we use a total of 20 different parameter pairs of tolerance loss to train the auxiliary network, and take the *δ* and *λ* pair with the best segmentation performance as the selected values of proposed tolerance loss.

When our method is applied to other different types of datasets of medical segmentation tasks or different segmentation models, the hyperparameter configurations of loss functions are different, and the hyperparameter values need to be redetermined. This is because the hyperparameter selection of the loss function needs to consider the imbalance of different datasets and the individual differences of attention maps generated by different models.

## 3. Experimental Results and Analysis

### 3.1. Dataset and Training

The ATLAS dataset has a high 3D resolution that can meet the requirements of rotation slicing operations, which contains 239 MRI data and focuses on the subacute and chronic stages of stroke disease. The operations of MNI-152 [24] image registration, intensity normalization [25], bias field correction [26], and changing the resolution of MRI scans to 176  × 208  ×  176 through cropping and interpolation operation to fit our method have been performed. We use the sixfold cross-validation to ensure that the test sets can cover the entire dataset. We also divide the training set of each fold into the inner loop training set and the inner loop validation set for best model selection. It should be noted that since the distribution of the number of MRIs of different sizes is extremely imbalanced in the dataset, it is necessary to ensure that the training, validation, and test sets have similar lesions sizes' distribution.

We use the deep learning framework PyTorch to conduct our experiments on three NVIDIA Tesla T4 GPUs. We train the models 100 epochs at most and save the best model when the validation set loss is the smallest. We used the lookahead optimizer [27] for model training. The optimizer improves the stability of the optimization process while considering the dynamic adjustment of the learning rate and the acceleration of the gradient descent. We set the initial learning rate to 1 × 10^−4^. The same experiment conditions and environment, used in the previous experiments in Section 2, are used for reproducing the single-path segmentation models, such as U-Net and attention U-Net. We applied the WBCE-Tversky loss for accurate segmentation to train these single-path models and use their results to compare the results of our DPAC-UNet method.

### 3.2. Experiment and Results

In Section 2.1, we elaborated on the principle of the proposed DPAC network structure. Using the attention U-Net as the basic segmentation model of the primary and auxiliary networks of the DPAC method, we proposed a specific segmentation model, DPAC-UNet. In Section 2.2, we also proposed the WBCE-Tversky loss and tolerance loss to train the primary and auxiliary networks, respectively. Moreover, we explored and verified the value of hyperparameter *β* of the WBCE-Tversky loss through the experiments presented in Tables 1 and 2 and found that when *β*=0.8, the primary network based on the attention U-Net achieves the best segmentation performance trained by the WBCE-Tversky loss.

We also explained the relationship between the values of different hyperparameters *δ* and *λ* and the coverage area of the auxiliary compensation attention coefficient map in Section 2.2. The coverage area of the auxiliary attention coefficient map is proportional to the FPR value, and the FPR value is proportional to *λ* and inversely proportional to *δ*. We need to select a suitable set of *λ* and *δ* values to obtain an auxiliary attention coefficient map with a suitable coverage area in order to enable the DPAC-UNet to achieve the best segmentation performance. Therefore, based on the experiment results, as presented in Table 3, we explored the optimal hyperparameter configuration of *λ* and *δ* to train the best DPAC-UNet model. We used the tolerance loss (*β*=0.8) configured with different hyperparameters *λ* and *δ* to train the auxiliary network of DPAC-UNet and the WBCE-Tversky loss (*β*=0.8) to train the primary network of the DPAC-UNet.

Table 4 presents the experiment results corresponding to the experiment of DPAC-UNet trained by the tolerance loss function with different hyperparameters. In Table 4, the FPR^*∗*^ represents the FPR results of single-path attention U-Net trained by tolerance loss functions with different hyperparameter configurations from Table 3. We sort FPR^*∗*^ in ascending order and identified the corresponding tolerance loss functions and hyperparameter configurations. We use tolerance loss functions with these sorted configurations to train the auxiliary network of the DPAC-UNet and the WBCE-Tversky loss (*β*=0.8) to train the primary network. Then, we got the experiment results of the different configurations of DPAC-UNet to select the best hyperparameter configuration.

By observing the relationship between FPR^*∗*^ and segmentation metrics, as presented in Table 4, it is evident that as the coverage area of the attention coefficient generated by the auxiliary network increases (indicated by FPR^*∗*^), the DSC and F2 scores of the DPAC-UNet gradually increase. When the values of the hyperparameters are *λ*=4 and *δ*=0.7, the DSC and F2 scores get the maximum value. As the FPR^*∗*^ further increases, the segmentation performance gradually declines. When the coverage area significantly increases with the FPR^*∗*^ value, it negatively affects the primary network. As presented in Figure 6, when *λ*=5 and *δ*=0.6, the FPR^*∗*^ value reaches the maximum, as well as the coverage area of the auxiliary compensation attention, which occupies a quarter of the brain slice. At this time, the coverage area is too large to constrain the primary network to focus on the correct lesion area effectively. Its attention coefficient map generated by this hyperparameter configuration even interferes with the primary network, so its DSC and F2 scores are negatively affected as presented in Table 4. The change of FPR^*∗*^ is determined by the hyperparameters *λ* and *δ* together. FPR^*∗*^ is proportional to *λ* and inversely proportional to *δ*. Therefore, the smallest *λ* and the largest *δ* will generate the smallest FPR^*∗*^, and the largest *λ* and smallest *δ*will lead to the largest FPR^*∗*^.  Figure 7 presents a line chart of the segmentation accuracy changing with FPR^*∗*^. The line chart indicates that the DPAC-UNet segmentation accuracy changes as the FPR^*∗*^ increases. As the FPR^*∗*^ increases, the DSC and F2 scores increase and then decrease. It shows that when the FPR^*∗*^ is small, the coverage area of the corresponding auxiliary attention compensation coefficient map is also small. It cannot compensate for the primary network adequately and effectively. When the FPR^*∗*^ value is too large, it tends to overcompensate. Only when the hyperparameter values are moderate and its corresponding FPR^*∗*^ value is moderate can the DPAC-UNet achieve the best segmentation performance.

Simultaneously, it can be seen from Table 4 that the FPR values generated by the DPAC-UNet's primary network are all small, irrespective of the loss function of the auxiliary network used and the corresponding FPR^*∗*^ value. This is because the compensation operation of the auxiliary compensation attention coefficient map generated by the auxiliary network does not directly affect the segmentation result of the primary network. It is an additive compensation operation from the auxiliary network to the primary network during the training process; therefore, it does not participate in the gradient operation and backpropagation of the primary network. However, it partially modified the size of the coverage area of the primary network's attention coefficient map. The primary network still considers accurate segmentation as its training purpose. It does not generate FP as high as the auxiliary network due to the increased attention area after compensation.

In summary, when the primary network uses the WCBE-Tversky loss function with hyperparameter configuration of *β*=0.8, and the auxiliary network uses tolerance loss function with hyperparameter configuration of *β*=0.8, *λ*=4, and *δ*=0.7, our DPAC-UNet can achieve the highest segmentation accuracy.

### 3.3. Visualization Examples

To show the principle of the DPAC-UNet, we give the attention coefficient heatmaps and segmentation results of using attention U-Net (primary network) individually and using DPAC-UNet with the auxiliary network when segmenting an MRI slice, as presented in Figure 8.

Using the primary network individually as presented in Figure 8(a), ② is the attention coefficient heatmap generated by the second-level AG of classic Attention U-Net; it can be observed that its attention coefficient map has obvious defects. Although the lesion's location is correct, the coverage area of the lesion is too small to perform accurate segmentation. ③ is the segmentation result; comparing ③ with the truth label of ①, it can be seen that there is a big difference between the segmentation result and the ground truth. When using the DPAC-UNet to segment the slice, as presented in Figure 8(b), ② is the attention coefficient heatmap generated by the primary network at the location marked as (I) in Figure 1. It is evident from the figure that the attention coefficient heatmap has obvious defects that are consistent with ②, as presented in Figure 8(a), which is also a defective attention heatmap with a smaller coverage area than the actual lesion. Notably, the attention coefficient heatmap ②, as presented in Figure 8(b), introduces a certain amount of noise. As presented in Figure 8(b), ③ is the auxiliary compensation attention coefficient generated by the DPAC-UNet's auxiliary network at the location marked as (II) in Figure 1. It is evident that the coverage area is moderately larger than the actual lesion, and covering the correct lesion region. After compensating the auxiliary compensation attention coefficient map of ③ to the primary network's attention coefficient map of ② through an additive compensation operation, a new attention coefficient map after compensation is obtained, as shown in ④. Comparing ④ and ②, as presented in Figure 8(b), the insufficient coverage area of attention coefficient in ② has been compensated, and the noise has also been significantly reduced. ⑤ is the final segmentation result of the DPAC-UNet. After using the DPAC-UNet, the segmentation result has been significantly improved in terms of both lesion contour and area. One thing to note here is when we compare the heatmap ② of Figure 8(a) generated by single-path attention U-Net and the heatmap ② of Figure 8(b) generated by DPAC-UNet's primary network, the attention heatmaps of Figures 8(a) and 8(b) are slightly different in noise level because they are two independent trained models, but the respective heatmap ② has the defects of the same pattern.

### 3.4. Comparison of Different Methods

Many lesion segmentation methods have been studied recently using the ATLAS dataset. Zhou et al. proposed a new architecture called dimension-fusion-UNet (D-UNet) [28], which combines 2D and 3D convolution in the encoding stage. Yang et al. proposed a CLCI-Net using cross-level fusion and a context inference network [29]. The previously mentioned existing segmentation results serve as a comparison for our experiments.

Using the same conditions as the previous experiments, we conducted a comparison experiment of the following models and loss functions:

1. the U-Net [9] model trained by the WBCE-Tversky loss (*β*=0.8)
2. the attention U-Net [10] trained by the WBCE-Tversky loss (*β*=0.8)
3. the DPAC-UNet model proposed in this paper, trained by the WBCE-Tversky loss and tolerance loss (*β*=0.8, *δ*=0.7, *λ*=4)

Cases (2) and (3) are, respectively, using the primary network individually and combined with the auxiliary network.

The final experiment comparison results are presented in Table 5 that the DPAC-UNet achieved the highest DSC and F2 scores. Comparing the single-path model attention U-Net with our DPAC-UNet, from using primary network individually to the introduction of the auxiliary attention compensation mechanism, the DSC score improved by 6%. Comparing the classic U-Net with attention U-Net, from no attention to the introduction of self-attention mechanism, the DSC score only improved by 2.1%. The previously mentioned comparison shows that our DPAC-UNet has a very significant performance improvement compared to the single-path self-attention segmentation model. Compared with the methods in the existing literature, it is 5.7% higher than the D-UNet and 1.1% higher than the CLCI-NET. This suggests that our DPAC-UNet achieved improved segmentation performance than the existing methods. As shown in Figure 9, we present a group of boxplots of the segmentation performance distribution of all 239 MRI scans to evaluate the performance of the different models. The 239 segmentation results are generated from the six nonrepeated test sets split by sixfold nested cross-validation. From the boxplots, we can state the following: first, comparing our DPAC-UNet model with the other two models, the overall segmentation accuracy increases significantly, and also, the minimum value of the boxplot of DSC and F2 scores and its lower quartile value increase significantly. This proves that our method significantly improves the data with poor performance using the other two methods. Second, when comparing the middle value and upper quartile of boxplots, we can see that, for the data with better segmentation performance segmented by the other two models, the DPAC-UNet has a slight improvement. For data with distinct lesion characteristics that are easy to segment, the primary network can generate a correct attention coefficient map with a high probability. At this time, using the auxiliary network to compensate the primary network will not reduce the segmentation accuracy or even slightly improve it. By observing the boxplots of the FPR results, it is evident that the FPR values of the three models are consistently small. This proves that although the auxiliary compensation attention coefficient map generated by the DPAC-UNet's auxiliary network has a high FPR, after compensating it to the primary network, the segmentation result of the primary network maintains a small FPR.

### 3.5. Time Consumption

The parameter amount, training, and testing computation time for each part of DPAC-UNet are listed in Table 6 to understand which part of the network needs more time for executing. Since the primary and auxiliary networks are trained in parallel as a whole, the computation time of each part cannot be measured separately at the same time. Therefore, we compared the computation complexity and time consumption of the primary and auxiliary networks of DPAC-UNet by training them independently.

The amount of our DPAC-UNet's training parameters is double compared with the single-path attention U-Net (primary network or auxiliary network). The training time of the DPAC-UNet (5.11 hours on average) is about 1.7 times that of each subnetwork (3.06 hours on average). The testing time of the DPAC-UNet (17 secs on average) is about 1.7 times that of each subnetwork (10 secs on average). Although DPAC-UNet has significantly increased the total number of model parameters and training time consumption after the introduction of the auxiliary network compensation mechanism, the significant improvement in segmentation performance makes up for the shortcoming of model complexity.

### 3.6. DPAC Structure of Other Models

The DPAC structure proposed in this paper that uses the auxiliary network to compensate the primary network can be applied to most segmentation models with spatial self-attention. We implemented our method on two other segmentation models with self-attention mechanism, RA-UNet [30] and AGResU-Net [31], and compared the experimental results of single-path with dual-path networks with auxiliary networks. The experimental results are shown in Table 7. The previously mentioned two single-path segmentation models can effectively improve the segmentation performance after using the auxiliary network for attention compensation. It shows that our method can be applied to other segmentation networks with the self-attention mechanism. It should be noted that, in accordance with the hyperparameter selection steps in Section 2.2.3, when the dataset and segmentation model change, the hyperparameters of the tolerance loss function need to be redetermined. As shown in Table 7, when the *δ* value of AGResU-Net is 0.6, the DPAC structure can achieve the best segmentation performance.

## 4. Discussion and Conclusions

In this paper, we proposed the DPAC-UNet using the classic self-attention model, attention U-Net, as the basic segmentation model. To realize the functions of the DPAC-UNet's primary and secondary networks, we proposed the WBCE-Tversky and tolerance losses as the training loss functions, respectively. We explored the hyperparameter configuration of the loss functions by applying sixfold cross-validation on the 239 MRI data of the ATLAS stroke segmentation dataset. We discovered that the WBCE-Tversky loss achieves the most accurate segmentation performance for the primary network when *β*=0.8. The tolerance loss generates a tolerant auxiliary compensation attention coefficient map with a moderate coverage area to compensate for the primary network's defective attention coefficient map. It achieves the best segmentation performance when *β*=0.8, *λ*=4, and *δ*=0.7. The experiment results indicate that the DSC score of the proposed DPAC-UNet with the auxiliary network is 6% higher than that without the auxiliary network. Compared with the methods in the existing literature, the DSC score of the proposed DPAC-UNet is 5.7% higher than the D-UNet and 1.1% higher than the CLCI-NET. The results indicate that the proposed method achieved an improved segmentation performance and verified the effectiveness of the proposed method.

It should be noted that although we used the same dataset in the proposed method as D-UNet and CLCI-NET, the version varied. We used the version without defacing that contains 239 MR images, and D-UNet and CLCI-NET used the version with defacing that contains 229 MR images. Furthermore, considering that the cross-validation dataset splitting methods do not generate the same training, validation, and testing sets, and also considering that the loss functions used are also different, achieving the best segmentation performance does not directly prove that the proposed method is the best. It proves that we have reached a higher level of segmentation performance in the current methods.

The purpose and focus of our work are to improve the performance of the single-path attention mechanism segmentation model by using our DPAC method. As shown in Table 6, although our method obviously requires more computing resources and takes more training time, the improvement in the segmentation performance of our method balances out the shortcomings in increased model complexity. The five-hour training time is currently at a lower or average level in some of the latest existing network models, which are currently used for stroke lesion segmentation. Moreover, we will implement our DPAC network structure on other basic segmentation models with a self-attention mechanism to verify our method's versatility. We also proved that if our DPAC structure is applied to other models based on the self-attention mechanism, it can also effectively improve the segmentation performance. In future work, we plan to use other stroke segmentation datasets to compare the effectiveness of our method across various datasets.

## Figures and Tables

**Figure 1:** Schematic of DPAC-UNet.

**Figure 2:** (a) Schematic of the AG structure of the auxiliary network, (b) schematic of the AG structure of the primary network, and (c) the definition of various operation symbols and dimensional changes of input and output feature signals.

**Figure 3:** Qualitative analysis of compensation mechanism of the auxiliary network.

**Figure 4:** Schematic of sixfold cross-validation.

**Figure 5:** Distribution of lesion volume in the training, test, and validation sets.

**Figure 6:** Attention coefficient heatmaps generated by the attention U-Net with different hyperparameters of the tolerance loss.

**Figure 7:** Segmentation performance of DPAC-UNet with the change in FPR^*∗*^.

**Figure 8:** Visualization examples of the attention coefficient maps of different methods: (a) single-path primary network individually; \(b) DPAC-UNet.

**Figure 9:** Boxplots of metric results for different models.

**Table 1:** Experimental results when using the Tversky loss with different *β* values to train the attention U-Net.

Weights	Metrics (%)			
	DSC	F2	PRE	RE
*α*=0.50, *β*=0.50	49.9	46.4	64.3	45.0
*α*=0.45, *β*=0.55	50.8	48.6	62.8	47.5
*α*=0.40, *β*=0.60	51.1	52.5	58.0	51.1
*α*=0.35, *β*=0.65	50.9	52.1	57.8	53.7
*α*=0.30, *β*=0.70	51.5	52.6	59.5	54.8
*α*=0.25, *β*=0.75	52.0	51.5	61.3	52.5
*α*=0.20, *β*=0.80	**52.7**	**55.4**	56.7	58.3
*α*=0.15, *β*=0.85	50.5	52.5	53.4	55.5
*α*=0.10, *β*=0.90	50.2	52.7	53.2	56.5
*α*=0.05, *β*=0.95	51.6	55.0	53.5	59.4

**Table 2:** Comparing the segmentation performance of the WBCE-Tversky loss under different hyperparameter configurations.

Loss functions	Weights	Metrics (%)				
		DSC	F2	PRE	RE	FPR
WBCE only	None	46.7	43.1	62.3	41.6	0.08
Tversky only	*α*=0.50, *β*=0.50	49.9	46.4	64.3	45.0	0.06
WBCE-Tversky		51.5	49.5	63.2	49.5	0.10
Tversky only	*α*=0.40, *β*=0.60	51.1	52.5	58.0	51.1	0.14
WBCE-Tversky		52.1	51.5	59.6	52.0	0.10
Tversky only	*α*=0.30, *β*=0.70	51.5	52.6	59.5	54.8	0.14
WBCE-Tversky		51.9	50.4	62.2	50.3	0.10
Tversky only	*α*=0.20, *β*=0.80	52.7	**55.4**	56.7	58.3	0.16
WBCE-Tversky		**53.2**	55.6	62.6	56.2	0.12
Tversky only	*α*=0.10, *β*=0.90	50.2	52.7	53.2	56.5	0.20
WBCE-Tversky		51.5	51.6	57.7	53.1	0.14

**Table 3:** FPR values of the tolerance loss using different hyperparameter configurations.

Loss functions	Weights		Metrics (%)				
			DSC	F2	PRE	RE	FPR
Tolerance loss *β* = 0.8	*λ*=1	*δ*=0.9	45.9	55.2	38.5	67.7	0.44
		*δ*=0.8	44.6	55.7	36.7	71.6	0.57
		*δ*=0.7	40.7	51.2	33.1	67.2	0.61
		*δ*=0.6	30.2	44.1	21.0	77.1	1.27
	*λ*=2	*δ*=0.9	45.2	55.4	36.3	70.6	0.51
		*δ*=0.8	32.2	45.3	23.0	72.6	1.09
		*δ*=0.7	30.4	44.6	20.6	70.9	1.34
		*δ*=0.6	14.8	26.0	8.9	83.5	4.44
	*λ*=3	*δ*=0.9	36.1	48.0	27.4	70.2	0.74
		*δ*=0.8	22.1	35.1	14.1	74.1	2014
		*δ*=0.7	22.8	36.1	14.8	79.4	2.01
		*δ*=0.6	11.8	18.8	7.6	83.5	4.57
	*λ*=4	*δ*=0.9	39.4	50.9	31.4	68.9	0.69
		*δ*=0.8	23.9	37.6	15.6	74.2	1.89
		*δ*=0.7	14.9	25.4	9.2	80.6	4.09
		*δ*=0.6	7.9	11.2	5.7	82.8	4.99
	*λ*=5	*δ*=0.9	34.4	47.5	24.9	72.4	0.90
		*δ*=0.8	20.7	33.5	13.3	82.3	2.74
		*δ*=0.7	13.2	24.1	7.8	84.1	5.63
		*δ*=0.6	5.7	11.8	3.1	92.8	**18.97**

**Table 4:** The segmentation performance of the DPAC-UNet using different hyperparameter configurations.

Loss functions	Weights		Metrics (%)					
			FPR^∗^	DSC	F2	PRE	RE	FPR
Tolerance loss, *β*=0.8	1.	*λ*=1, *δ*=0.9	0.438	54.8	54.1	63.6	55.1	0.111
	2.	*λ*=2, *δ*=0.9	0.508	53.0	52.4	61.5	53.3	0.101
	3.	*λ*=1, *δ*=0.8	0.573	55.2	54.7	64.4	55.7	0.120
	4.	*λ*=1, *δ*=0.7	0.607	54.1	54	62.2	55.1	0.117
	5.	*λ*=4, *δ*=0.9	0.689	55.9	56.6	63	57.4	0.124
	6.	*λ*=3, *δ*=0.9	0.743	55.3	56	61.1	58.1	0.173
	7.	*λ*=5, *δ*=0.9	0.898	53.8	54.1	62.8	55.7	0.142
	8.	*λ*=2, *δ*=0.8	1.091	54.9	55.4	61.2	56.9	0.140
	9.	*λ*=1, *δ*=0.6	1.27	55.5	55.6	63.7	57	0.126
	10.	*λ*=2, *δ*=0.7	1.335	55.8	55.8	64.8	57.2	0.133
	11.	*λ*=4, *δ*=0.8	1.888	53.6	53	64.4	53.9	0.111
	12.	*λ*=3, *δ*=0.7	2.006	56.9	57.7	61.6	59.6	0.149
	13.	*λ*=3, *δ*=0.8	2.143	56.7	57.3	61.9	59.1	0.157
	14.	*λ*=5, *δ*=0.8	2.744	56.7	56	65.8	56.8	0.103
	15.	*λ*=4, *δ*=0.7	**4.093**	**59.3**	**59.8**	65.6	59.9	0.106
	16.	*λ*=2, *δ*=0.6	4.44	58.2	58.6	62.6	60.3	0.151
	17.	*λ*=3, *δ*=0.6	4.57	57.5	57.5	64	58.8	0.137
	18.	*λ*=4, *δ*=0.6	4.99	56.5	56.9	62.5	61.6	0.153
	19.	*λ*=5, *δ*=0.7	5.634	56.2	57.5	63	59.3	0.132
	20.	*λ*=5, *δ*=0.6	18.97	52.8	51.5	65.9	52.1	0.196

**Table 5:** Comparison of segmentation performance of different methods.

Models	Loss functions	Metrics (%)			
		DSC	F2	PRE	RE
D-UNet	Enhance mixing loss	53.5	—	63.3	52.4
CLCI-NET	Dice loss	58.1	—	64.9	58.1
U-Net	WBCE-Tversky(*β*=0.8)	51.1	49.2	59.3	48.7
Attention U-Net	WBCE-Tversky(*β*=0.8)	53.2	55.6	62.6	56.2
DPAC-UNet	WBCE-Tversky(*β*=0.8), tolerance(*δ*=0.7, *λ*=4)	**59.2**	**59.0**	**65.6**	**59.9**

**Table 6:** Time consumption of DPAC-UNet.

Networks	Parameters (M)	Training (hours)	Testing (seconds)
Primary network	40.4	3.07	10
Auxiliary network	40.4	3.05	10
DPAC-UNet	80.8	5.11	17

**Table 7:** Experimental results of DPAC structure based on other models.

No.	Networks	Auxiliary	Loss functions	Metrics (%)			
				DSC	F2	PRE	RE
1	RA-UNet	Without	WBCE-Tversky (*β*=0.8)	54.1	56.5	63.8	58.1
		With	WBCE-Tversky (*β*=0.8), tolerance (*δ*=0.7, *λ*=4)	**60.3**	**59.9**	**67.1**	**60**
2	AGResU-Net	Without	WBCE-Tversky (*β*=0.8)	55.2	59.7	61.4	57.5
		With	WBCE-Tversky (*β*=0.8), tolerance (*δ*=0.6, *λ*=4)	**60.5**	**62.2**	**66.6**	**61.1**

## Data Availability

The ATLAS dataset is publicly available at http://fcon_1000.projects.nitrc.org/indi/retro/atlas_download.html.

## References

[1] Thrift A. G., Cadilhac D. A., Thayabaranathan T. (2014). Global stroke statistics. *International Journal of Stroke*.

[2] Zhang R., Zhao L., Lou W. (2018). Automatic segmentation of acute ischemic stroke from DWI using 3-D fully convolutional DenseNets. *IEEE Transactions on Medical Imaging*.

[3] Liew S. L., Anglin J. M., Banks N. W. (2018). A large, open source dataset of stroke anatomical brain images and manual lesion segmentations. *Scientific data*.

[4] LeCun Y., Bottou L., Bengio Y., Haffner P. (1998). Gradient-based learning applied to document recognition. *Proceedings of the IEEE*.

[5] Shelhamer E., Long J., Darrell T. (2017). Fully convolutional networks for semantic segmentation. *IEEE Transactions on Pattern Analysis and Machine Intelligence*.

[6] Badrinarayanan V., Kendall A., Cipolla R. (2017). SegNet: a deep convolutional encoder-decoder architecture for image segmentation. *IEEE Transactions on Pattern Analysis and Machine Intelligence*.

[7] Suzuki K. (2017). Overview of deep learning in medical imaging. *Radiological Physics and Technology*.

[8] Litjens G., Kooi T., Bejnordi B. E. (2017). A survey on deep learning in medical image analysis. *Medical Image Analysis*.

[9] Ronneberger O., Fischer P., Brox T. U-net: convolutional networks for biomedical image segmentation.

[10] Schlemper J., Oktay O., Schaap M. (2019). Attention gated networks: learning to leverage salient regions in medical images. *Medical Image Analysis*.

[11] Zhou Z., Siddiquee M. M. R., Tajbakhsh N., Liang J. UNet++: a nested U-net architecture for medical image segmentation.

[12] Alom M. Z., Yakopcic C., Taha T. M., Asari V. K. Nuclei segmentation with recurrent residual convolutional neural networks based U-Net (R2U-Net).

[13] Lin B. S., Michael K., Kalra S., Tizhoosh H. R. Skin Lesion Segmentation: U-Nets versus Clustering.

[14] Noori M., Bahri A., Mohammadi K. Attention-guided version of 2D UNet for automatic brain tumor segmentation.

[15] Huang Y. J., Dou Q., Wang Z. X. (2020). 3-D RoI-aware U-net for accurate and efficient colorectal tumor segmentation. *IEEE Transactions on Cybernetics*.

[16] Christ P. F., Elshaer M. E. A., Ettlinger F. Automatic liver and lesion segmentation in CT using cascaded fully convolutional neural networks and 3D conditional random elds.

[17] Sirinukunwattana K., Pluim J. P. W., Chen H. (2017). Gland segmentation in colon histology images: the glas challenge contest. *Medical Image Analysis*.

[18] Çiçek Ö., Abdulkadir A., Lienkamp S. S., Brox T., Ronneberger O. 3D U-net: learning dense volumetric segmentation from sparse annotation.

[19] Merkow J., Marsden A., Kriegman D., Tu Z. Dense volume-to-volume vascular boundary detection.

[20] Khened M., Kollerathu V. A., Krishnamurthi G. (2019). Fully convolutional multi-scale residual DenseNets for cardiac segmentation and automated cardiac diagnosis using ensemble of classifiers. *Medical Image Analysis*.

[21] Li Y., Shen L. Deep learning based multimodal brain tumor diagnosis.

[22] Salehi S. S. M., Erdogmus D., Gholipour A. Tversky loss function for image segmentation using 3D fully convolutional deep networks.

[23] Sudre C. H., Li W., Vercauteren T., Ourselin S., Jorge Cardoso M. (2017). Generalised dice overlap as a deep learning loss function for highly unbalanced segmentations. *Deep Learning in Medical Image Analysis and Multimodal Learning for Clinical Decision Support*.

[24] Collins D. L., Neelin P., Peters T. M., Evans A. C. (1994). Automatic 3D intersubject registration of MR volumetric data in standardized Talairach space. *Journal of Computer Assisted Tomography*.

[25] Sled J. G., Zijdenbos A. P., Evans A. C. (1998). A nonparametric method for automatic correction of intensity nonuniformity in MRI data. *IEEE Transactions on Medical Imaging*.

[26] Tustison N. J., Avants B. B., Cook P. A. (2010). N4ITK: improved N3 bias correction. *IEEE Transactions on Medical Imaging*.

[27] Zhang M., Lucas J., Ba J., Hinton G. E. Lookahead Optimizer: k steps forward, 1 step back.

[28] Zhou Y., Huang W., Dong P., Xia Y., Wang S. (2021). D-UNet: a dimension-fusion U shape network for chronic stroke lesion segmentation. *IEEE/ACM Transactions on Computational Biology and Bioinformatics*.

[29] Yang H., Huang W., Qi K. CLCI-net: cross-level fusion and context inference networks for lesion segmentation of chronic stroke.

[30] Jin Q., Meng Z., Sun C., Cui H., Su R. (2020). RA-UNet: A hybrid deep attention-aware network to extract liver and tumor in CT scans. *Frontiers in Bioengineering and Biotechnology*.

[31] Zhang J., Jiang Z., Dong J., Hou Y., Liu B. (2020). Attention gate resU-Net for automatic MRI brain tumor segmentation. *IEEE Access*.

